The article "Risk Factors for Brain Metastasis of Hepatocellular Carcinoma" was retracted in 2023. Reasons: unreliable results or conclusions; concerns about the data; concerns about the peer review; concerns about the citations.

# Risk Factors for Brain Metastasis of Hepatocellular Carcinoma

**DOI:** 10.1155/2022/7848143

**Published:** 2022-03-09

**Authors:** Lei Wang, Yongze Guo, Hongwei Zhang, Hua Li, Fei Wang, Jiuna Zhang, Xiaotian Li

**Affiliations:** ^1^Department of Gastroenterology, Affiliated Hospital of Hebei Engineering University, Handan 056002, China; ^2^Department of Infectious Diseases, Affiliated Hospital of Hebei Engineering University, Handan 056002, China; ^3^Department of Endocrinology, Handan HanGang Hospital, Hebei Province, Handan 056004, China

## Abstract

Hepatocellular carcinoma (HCC) is a common malignancy with high mortality, especially in HCC patients with brain metastases (BMS). However, few studies have investigated the risk factors for BMS among HCC patients based on large-scale population. The study involved clinical data of 36,091 patients who met the inclusion criteria from the SEER database, from 2004 to 2016. Univariate analysis and multifactor logistics regression analysis was used to analyze risk factors affecting BMS among HCC patients. This study revealed that BMS occurred in 108 of 36,091 patients, with an incidence of 0.33%. Median survival was 7 months for patients with BMS, but 12 months for patients without BMS. Univariate analysis showed that pathological low differentiation and undifferentiation, lymph node metastasis, no surgical treatment, and no chemotherapy and radiotherapy increased risk of BMS (*P* < 0.05). Multivariate analysis suggested that no surgical treatment and no chemotherapy or radiotherapy were independent risk factors for BMS (*P* < 0.001). Our findings highlighted that the independent risk factors for BMS were no surgical treatment, no chemotherapy, and no radiotherapy.

## 1. Introduction

Hepatocellular carcinoma (HCC) is the fifth most common malignant tumor in the world, with about 800,000 new cases every year [1, 2]. HCC has a poor prognosis, with a 5-year overall survival of 18%, especially for patients with brain metastases, with a median OS of 1.2–2.4 months [3, 4] and a very high mortality rate. However, due to the low incidence of HCC with BMS, overall accounting for 0.2%–2.2% [5], poor prognosis, and lack of specific symptoms of early BMS, clinicians rarely pay attention to HCC.

BMS from HCC usually occurs 18–31 months after the initial diagnosis of HCC. Due to the difficulty of early diagnosis of BMS, and HCC patients often spread to other extrahepatic sites before BMS, the indications for the treatment of HCC patients with BMS are a major challenge for surgeons. Early diagnosis of BMS, radiotherapy combined with molecular targeted therapy and immunotherapy, can bring certain treatment opportunities for advanced HCC patients with BMS [5–7].

It is of practical clinical significance to screen out high-risk HCC patients with BMS rapidly through simple clinical data and then conduct relatively accurate early screening. This study's main aim is to use the Surveillance, Epidemiology, and End Results (SEER) database to describe the incidence of BMS in HCC patients at the time of cancer diagnosis at a population level and to explore the risk factors related to HCC brain metastases, providing reference for the diagnosis and treatment of HCC brain metastases.

## 2. Materials and Methods

### 2.1. Patients

The study involved a retrospective evaluation of medical records from the Surveillance, Epidemiology, and End Results (SEER) program (http://www.seer.cancer.gov), the SEER*∗*Stat database, with cancer patient data registered since 1973. In this study, SEER Stat software (8.3.6) was used to retrieve 75,706 patients over 18 years of age who were pathologically diagnosed with HCC from 2004 to 2016. Inclusion criteria were as follows: (1) patients whose pathology diagnosed as HCC; (2) patient aged 18 years or older; (3) patients with complete follow-up data. Exclusion criteria were as follows: (1) patient's history of brain metastases is unknown; (2) patients with incomplete follow-up data; (3) patients with two or more primary malignancies. Patients who met the inclusion and exclusion criteria were screened, and the detailed data screening process is shown in Figure 1. The patients with brain metastases were diagnosed the by the specific ICD codes in the SEER database.

### 2.2. Data Collection

Patients' clinical data were obtained from the SEER database and screened according to inclusion criteria, followed by further statistical analysis. The variables were selected to identify the risk factors of BMS in HCC patients are as follows: age at diagnosis, sex, race, important clinical pathological information, including primary tumor size, grade, AFP, degree of liver fibrosis, N-stage according to the version 7 AJCC staging system, vascular invasion, and the treatment information including surgery, radiotherapy, and chemotherapy.

### 2.3. Statistical Analysis

All of the statistical analyses were conducted with SPSS Statistics (version 22.0) as well as the SEER*∗*Stat program (version 8.3.6). Kaplan–Meier (K–M) analysis was used to compare the overall survival (OS) of patients. In addition, the risk factors of classification variables for univariate analysis were identified using the Chi-square test. Statistical significance was declared with a two-sided *p* value <0.05.

## 3. Results

### 3.1. Baseline Characteristics of Patients

A total of 36091 HCC patients whose records were extracted from the SEER database were included. Figure 1 shows the flow chart. Of these patients, about 120 (70.45%) showed brain metastases. In the cohort, 77.49% of patients were male, mostly white (68.31%) and AFP positive (59.37). The median overall survival (mOS) of patients without BMS was 12 months (95% CI (11.669, 12.331)), while that of patients with BMS was only 7 months (95% CI (4.344, 9.656)), which was significantly lower than that of patients without BMS (*P* = 0.024).  Table 1 shows the baseline characteristics of the included patients.

### 3.2. Univariate Analysis of Risk Factors for Developing BMS

Table 2 and 3 show the univariate analysis. The patients with lower grade, metastasis of undifferentiated lymph nodes, no surgical resection, no chemotherapy, and no radiotherapy were likely to have brain metastases, when univariate analysis was performed to evaluate the risk of brain metastases in HCC patients based on age, sex, and clinical data.

### 3.3. Multivariate Logistic Regression Analysis of Risk Factors for Developing BMS

Table 4 shows the multivariate analysis, and the variables with *P* value < 0.05 in univariate analysis were included in multivariate logistic regression analysis to determine the risk factors of HCC with BMS. The variables included tumor differentiation degree, lymph node metastasis, surgical history, and history of radiotherapy and chemotherapy. The grade of tumor differentiation was excluded from the stepwise forward regression analysis. The results showed that the absence of surgery, chemotherapy, and radiotherapy were independent risk factors for BMS (*P* < 0.001).

## 4. Discussion

Presently, the prognosis of HCC remains poor, especially for patients with advanced HCC, whose 5-year survival rate is only around 3.1% [8]. Patients with HCC complicated with BMS had a worse prognosis, with a median survival time of 7 months in this study. At present, many studies had been devoted to exploring the prognostic factors of HCC complicated with BMS [9, 10]. A study in China has explored the risk factors and prognostic factors of HCC with lung metastasis through the SEER database [11]. However, there is still a lack of large clinical data to support the epidemiological characteristics of HCC with BMS. This study analyzed the incidence of BMS in HCC patients and explored its risk factors.

The incidence of BMS from HCC was the highest in patients with undifferentiated tumors and patients receiving radiotherapy, which were 0.92% and 2.18%, respectively. Undifferentiated HCC was highly malignant and was prone to brain metastasis. Radiotherapy is an effective treatment for inoperable HCC. The results of a research which performed radiotherapy on 115 HCC patients showed that 40% of the patients reached CR and 88.7% of the patients had PR [12], but the reason why brain metastases were more likely to occur in the patients who received radiotherapy was not yet clear. A number of studies have found that radiotherapy also plays an important role in promoting tumor metastasis. Some researchers have found that, during radiotherapy, dying prostate cancer cells mediate TLR2 receptors and activate the PI3K/pAKT pathway to promote the metastasis of surviving tumor cells [13]. In addition, the changes in the tumor microenvironment caused by radiotherapy may lead to local hypoxia, thereby increasing the tumor's invasion and metastasis ability [14]. It can be seen that, in addition to its therapeutic effects, radiotherapy may also cause changes in the biological behavior of residual tumor cells. The mechanism needs more evidence to support.

The present study showed that, in addition to tumor differentiation and radiotherapy history, patients with lymph node metastasis, surgery, or chemotherapy were risk factors for BMS in HCC patients. Patients with high levels of AFP and poorly differentiated tumors were more malignant and more aggressive [7]. Moderately poorly differentiated and undifferentiated tumors are prone to brain metastasis, but alpha-fetoprotein has no obvious effect. This may be related to the specific quantitative level of AFP, and further research is needed. In addition, general conditions such as age, gender, race, marital status, and clinical information such as tumor size, vascular invasion, and degree of liver fibrosis also did not have a significant impact on the occurrence of brain metastases (*P* > 0.05). The data were further analyzed by multivariate logistic regression analysis. As shown in Table 2, no surgery, no history of chemotherapy, and history of radiotherapy were independent risk factors for brain metastasis in HCC patients. Patients who have not undergone surgery or chemotherapy or received radiotherapy were more likely to have brain metastases. Early surgery or chemotherapy for HCC patients who met the indications may reduce the occurrence of liver cancer brain metastases.

Although this study comprehensively analyzed the risk factors for brain metastases in HCC patients, it still has its shortcomings. First of all, this study only obtained information on whether brain metastases exist at the time of HCC diagnosis, but the SEER database did not provide the characteristics of disease recurrence or the disease that occurred during follow-up, and it is difficult to evaluate the occurrence of brain metastases during treatment. Therefore, there might be some patients with brain metastases in the later stages of the disease, but relevant information was not available. Future studies may be able to use data from other sources to solve this important problem. Secondly, patients with HCC were not routinely screened by enhanced MRI of the brain. Many patients were only discovered because of their brain metastases. Therefore, this study might underestimate the incidence of HCC brain metastases. The incidence of brain metastases in patients without neurological symptoms was currently unclear. The SEER database did not record detailed radiotherapy and chemotherapy related data, and different chemotherapy drugs might affect the efficacy. In addition, the specific site of radiotherapy or the time point of radiotherapy selection was not clearly stated. In this study, patients with radiotherapy had the highest incidence of brain metastases, whether it was also possible that patients with brain metastases had more opportunities to receive radiotherapy. Therefore, the impact of radiotherapy on the incidence of HCC brain metastasis requires more detailed treatment data to analyze.

In conclusion, despite these limitations, this study conducted an in-depth study of the epidemiological characteristics of HCC patients with brain metastases. No surgery, no history of chemotherapy, and history of radiotherapy are independent risk factors for brain metastasis in HCC patients. This study can guide patients with high-risk brain metastases from liver cancer to undergo brain-enhanced MRI examinations, early diagnosis, and treatment to prolong the survival of patients. In view of the deficiencies in this study, more clinical data are needed for further exploration.

## Figures and Tables

**Figure 1:** The flow chart of the study.

**Table 1:** The baseline characteristics of the included patients.

Variables	Patients
Age	
<65	21445
≥65	14646
Race	
Black	5106
White	24653
Others	6104
Sex	
Male	27967
Female	8124
Marital status	
Married	17274
Unmarried	8252
Others	10565
Tumor size	
≤3 cm	8697
>3 and ≤5 cm	6560
>5 cm	11076
AFP	
Positive	21427
Negative	7609
Others	7055
Vascular invasion	
Yes	5366
No	17029
Unknown	13696
Fibrosis degree	
F0	1763
F1	8789
Unknown	25539
N stage	
N0	26167
N1	2223
Unknown	7701
Differentiated degree	
High differentiation	3438
Moderately differentiated	5437
Low differentiated	2546
Undifferentiation	217
Unknown	24453
Radiotherapy	
Yes	411
No	35680
Chemotherapy	
Yes	15311
No	20780
Surgery	
Yes	8349
No	27348
Unknown	404

**Table 2:** Univariate analysis of baseline risk factors for HCC brain metastases.

Variables	Non-BMS, *n* (%)	BMS, *n* (%)	*p* value
Age			0.780
<65	21372 (99.7)	73 (0.3)	
≥65	14599 (99.7)	47 (0.3)	
Race			0.347
Black	5084 (99.6)	22 (0.4)	
White	24573 (99.7)	80 (0.3)	
Others	6087 (99.7)	17 (0.3)	
Sex			0.516
Male	27871 (99.7)	96 (0.3)	
Female	8100 (99.7)	24 (0.3)	
Marital status			0.929
Married	17218 (99.7)	56 (0.3)	
Unmarried	8225 (99.7)	27 (0.3)	
Others	10528 (99.7)	37 (0.3)	

**Table 3:** Univariate analysis of cancer-related risk factors for HCC brain metastases.

Variables	Non-BMS, *n* (%)	BMS, *n* (%)	*p* value
Tumor size			0.070
≤3 cm	8681 (99.8)	16 (0.2)	
>3 and ≤5 cm	6549 (99.8)	11 (0.2)	
>5 cm	11041 (99.7)	35 (0.3)	
AFP			0.090
Positive	21355 (99.7)	72 (0.3)	
Negative	7593 (99.8)	16 (0.2)	
Others	7023 (99.6)	32 (0.4)	
Vascular invasion			0.348
Yes	5356 (99.8)	10 (0.2)	
No	16984 (99.7)	45 (0.3)	
Unknown	13631 (99.5)	65 (0.5)	
Fibrosis degree			0.939
F0	1758 (99.7)	5 (0.3)	
F1	8765 (99.7)	24 (0.3)	
Unknown	25448 (99.6)	91 (0.4)	
N stage			0.035
N0	26101 (99.8)	66 (0.0)	
N1	2212 (99.5)	11 (0.5)	
Unknown	7658 (99.4)	43 (0.6)	
Differentiated degree			0.020
High differentiation	3432(99.8)	6 (0.2)	
Moderately differentiated	5419 (99.7)	18 (0.3)	
Low differentiated	2531 (99.4)	15 (0.6)	
Undifferentiation	215 (99.1)	2 (0.9)	
Unknown	24374 (99.7)	79 (0.3)	
Radiotherapy			<0.001
Yes	402 (97.8)	9 (2.2)	
No	35569 (99.7)	111 (0.3)	
Chemotherapy			<0.001
Yes	15282 (99.8)	29 (0.2)	
No	20689 (99.6)	91 (0.4)	
Surgery			<0.001
Yes	8344 (99.9)	5 (0.1)	
No	27223 (99.6)	115 (0.4)	
Unknown	404 (100)	0	

**Table 4:** Multivariate logistic analysis of risk factors for HCC brain metastases.

Variables	OR (95% CI)	*p* value
N stage		
N0	Reference	NA
N1	1.43 (0.75,2.74)	0.270
Unknown	1.90 (1.29,2.79)	0.011
Radiotherapy		
Yes	23.15 (10.95,48.94)	<0.001
No	Reference	NA
Chemotherapy		
Yes	Reference	NA
No	2.56 (1.68,3.90)	<0.001
Surgery		
Yes	Reference	NA
No	12.65 (4.87,32.84)	<0.001
Unknown	<0.001	0.995

## Data Availability

The simulation experiment data used to support the findings of this study are available from the corresponding author upon request.
